# The Role of Neurotrophin-4/Forkhead Box L1 in the Development of Nonsmall-Cell Lung Cancer

**DOI:** 10.1155/2022/9078012

**Published:** 2022-08-09

**Authors:** Lin Mu, Hong Zhao, Yifeng Zhang, Chun Xiao

**Affiliations:** ^1^Department of Pulmonary and Critical Care Medicine, Heping Hospital Affiliated to Changzhi Medical College, Changzhi, China; ^2^Department of General Surgery, PLA Rocket Force Characteristic Medical Center, Beijing, China

## Abstract

This study aims to uncover the biological function of neurotrophin-4 (NTF4) in affecting the progression of nonsmall-cell lung cancer (NSCLC). NTF4 levels in NSCLC and paracancerous tissues were detected by quantitative real-time polymerase chain reaction (qRT-PCR). Knockdown of NTF4 in A549 and H1299 cells was achieved by transfection of sh-NTF4. Subsequently, proliferative and migratory changes in NSCLC cells with NTF4 knockdown were determined by cell counting kit-8 (CCK-8) and transwell and wound healing assay. The target gene binding NTF4 was predicted by bioinformatic software and verified by a dual-luciferase reporter assay. The role of the NTF4/FOXL1 axis in mediating NSCLC cell behaviors was finally explored through rescue experiments. NTF4 was highly expressed in NSCLC tissues than in normal ones. Knockdown of NTF4 remarkably reduced proliferative and migratory rates in A549 and H1299 cells. Forkhead Box L1 (FOXL1) was confirmed as a target gene of NTF4 by bioinformatic software and verified by a dual-luciferase reporter assay. Knockdown of FOXL1 was able to reverse the reduced proliferative and migratory rates in A549 and H1299 cells transfected with sh-NTF4. NTF4 triggers NSCLC to proliferate and migrate via negatively regulating FOXL1.

## 1. Introduction

Lung carcinoma is the malignant tumor with the highest incidence in the world. In 2018, lung carcinoma patients account for 20.27% and 12.59% of all male and female cancer cases, respectively [1, 2]. NSCLC is the main subtype of lung carcinoma, including squamous cell carcinoma and adenocarcinoma [3, 4]. Seriously, the 5-year survival of nonsmall-cell lung cancer (NSCLC) is less than 15%, even for patients who received active treatments [5, 6]. At present, diagnostic and therapeutic targets for NSCLC are lacking, and great efforts should be made on seeking for effective biomarkers [7, 8].

NTF4 is a newly discovered pathogenic gene [9, 10]. NTF4 protein can activate the tyrosine kinase-B receptor (TrkB) and prevents against ocular hypertension, ischemia, and release of cytotoxins [11]. In addition, NTF4 variation impairs TrkB signaling, thus affecting the growth of tumor cells [11, 12]. NTF4 was also reported to be upregulated in gastric cancer tissues and predicted poor overall survival and progression-free survival in GC patients [13]. Therefore, it is believed that NTF4 variation is of significance in the tumor process. Through literature review, NTF4 is able to aggravate the malignant progression of colorectal carcinoma [9, 14].

With the rapid development of molecular biology, the complicated network involving NTF4 and its downstream target is conductive to provide novel strategies for clinical treatment of NSCLC. This study first detected differential levels of NTF4 in NSCLC samples and later explored its biological functions in mediating malignant phenotypes of NSCLC and the underlying molecular mechanism.

## 2. Methods

### 2.1. NSCLC Samples

A total of 19 pairs of NSCLC and adjacent normal tissues were collected from surgery, puncture biopsy, or bronchoscopy biopsy. Adjacent tissues were at least 5 cm away from tumor lesions. None of the recruited patients had preoperative chemotherapy or radiotherapy. This study was approved by the research ethics committee of our hospital and complied with the Helsinki Declaration. Informed consent was obtained from patients.

### 2.2. Cell Lines and Reagents

NSCLC cell lines (A549, H1299, PC-9, H358, and SPC-A1) and the human bronchial epithelial cell line (BEAS-2B) were purchased from American Type Culture Collection (ATCC) (Manassas, VA, USA). Cells were cultured in Dulbecco's modified eagle medium (DMEM) containing 10% fetal bovine serum (FBS) at 37°C with 5% CO_2_ (Gibco, Rockville, MD, USA).

### 2.3. Transfection

Transfection plasmids were synthesized by GenePharma (Shanghai, China). Cells were cultured to 40–60% density in a 6-well plate and transfected using Lipofectamine 2000 (Invitrogen, Carlsbad, CA, USA). After 48 h cell transfection, cells were collected for verifying transfection efficacy and functional experiments.

### 2.4. Cell Counting Kit-8 (CCK-8) Assay

Cells were inoculated in a 96-well plate with 2 × 10^3^ cells/well. At 24, 48, 72, and 96 h, optical density at 450 nm of each sample was recorded using the CCK-8 kit (Dojindo Laboratories, Kumamoto, Japan) for plotting the viability curves.

### 2.5. Transwell Assay

The cell suspension was prepared at 5 × 10^5^ cells/mL. 200 *μ*L of suspension and 700 *μ*L of medium containing 20% FBS were, respectively, added to the top and bottom of a transwell insert, and cultured for 48 h. Cells were migrated from the top to the bottom, which were induced with methanol for 15 min, 0.2% crystal violet for 20 min, and captured using a microscope. Five random fields per sample were selected for capturing and counting cells.

### 2.6. Wound Healing Assay

Cell suspension in serum-free medium was prepared at 5 × 10^5^/mL and implanted in 6-well plates. Cells were cultivated to 90% density, followed by creating an artificial scratch using a sterilized pipette tip. Cells were washed in phosphate-buffered saline (PBS) for 2-3 times and cultured in the medium containing 1% FBS. 24 hours later, the wound closure percentage was calculated.

### 2.7. Quantitative Real-Time Polymerase Chain Reaction (qRT-PCR)

Cells were lysed using TRIzol reagent (Invitrogen, Carlsbad, CA, USA) for isolating RNAs. Qualified RNAs were reversely transcribed into complementary deoxyribose nucleic acids (cDNAs) using the AMV reverse transcription kit (TaKaRa, Otsu, Japan), followed by qRT-PCR using StepOnePlus Real-Time PCR (Applied Biosystems, CA, USA). Glyceraldehyde-3-phosphate dehydrogenase (GAPDH) was the internal reference. Each sample was performed in triplicate, and the relative level was calculated by 2^−ΔΔCt^. NTF4: forward: 5′-AGATGTCAGGAAGGAGGGGG-3′, reverse: 5′-CATCTCTCGGAGCACCTGTC-3′; FOXL1: forward: 5′-TTCAACGCTTCCCTGATGCT-3′, reverse: 5′-GAACCGTGCCATTGTTTGCT-3′; and GAPDH: forward: 5′- GGAGCGAGATCCCTCCAAAAT -3′, reverse: 5′- GGCTGTTGTCATACTTCTCATGG -3′.

### 2.8. Western Blot

Cells were lysed in radioimmunoprecipitation assay (RIPA) (Beyotime, Shanghai, China) on ice for 15 min, and the mixture was centrifuged at 14000 × g, 4°C for 15 min. The concentration of cellular protein was determined by the bicinchoninic acid (BCA) method (Pierce, Rockford, IL, USA). Protein samples with the adjusted same concentration were separated by sodium dodecyl sulfate-polyacrylamide gel electrophoresis (SDS-PAGE) and loaded on polyvinylidene fluoride (PVDF) membrane (Millipore, Billerica, MA, USA). The membrane was cut into small pieces according to the molecular size and blocked in 5% skim milk for 2 h. They were incubated with primary and secondary antibodies, followed by band exposure and gray value analyses using alpha SP. Rabbit monoclonal NTF4 antibody (dilution: 1/500; CatNo: ab150437), rabbit polyclonal GAPDH antibody (dilution: 1 : 500, CatNo: ab37168), and secondary goat anti-rabbit (HRP) IgG antibody (dilution: 1/2000; CatNo: ab6721) were all purchased from Abcam (Cambridge, MA, USA).

### 2.9. Dual-Luciferase Reporter Assay

Cells were seeded in a 24-well plate, which were cotransfected with pcDNA-FOXL1/pcDNA-NC and pmirGLO-NTF4-WT/pmirGLO-NTF4-MUT, respectively. Luciferase activity (Promega, Madison, WI, USA) was measured at 48 h in a standard method.

### 2.10. Statistical Analysis

GraphPad Prism 5 V5.01 (La Jolla, CA, USA) was used for statistical analyses, and data were expressed as mean ± standard deviation. Differences between groups were compared by the *t*-test. Potential influences of NTF4 and FOXL1 on NSCLC pathology were analyzed by the chi-square test. *P* < 0.05 was considered statistically significant.

## 3. Results

### 3.1. NTF4 Was Highly Expressed in NSCLC

Differential levels of NTF4 were detected in 19 pairs of NSCLC and adjacent normal tissues. As qRT-PCR data revealed, NTF4 was upregulated in NSCLC tissues (Figures 1(a) and 1(b)). Besides, NTF4 was highly expressed in NSCLC cell lines (Figure 1(c)).

### 3.2. Knockdown of NTF4 Reduced Proliferative and Migratory Rates in NSCLC

Transfection efficacy of sh-NTF4 was examined in A549 and H1299 cells by Western blot (Figure 2(a)). CCK-8 assay revealed a reduction in cell viability after transfection of sh-NTF4 in A549 and H1299 cells, suggesting the inhibited proliferative potential (Figures 2(b) and 2(c)). In addition, declined migratory cell number and wound closure percentage owing to knockdown of NTF4 in NSCLC cells indicated that NTF4 stimulated migratory ability (Figures 2(d) and 2(e)).

### 3.3. NTF4 Targeted the Regulation of FOXL1

A potential interaction between NTF4 and FOXL1 was predicted using bioinformatic tools (Figure 3(a)). Subsequently, overexpression of FOXL1 was detected to reduce luciferase activity in pmirGLO-NTF4-WT, while it had no impact on luciferase activity in pmirGLO-NTF4-MUT (Figures 3(b) and 3(c)). It is suggested that NTF4 could be targeted by FOXL1 through the predicted binding site. Compared with normal tissues, FOXL1 was lowly expressed in NSCLC tissues (Figures 3(d) and 3(e)).

### 3.4. NTF4-Regulated NSCLC Cell Phenotypes by Negatively Regulating FOXL1

A series of rescue experiments were conducted to analyze the involvement of FOXL1 in NTF4-regulated NSCLC cell phenotypes. Transfection efficacy of sh-FOXL1 was examined in A549 and H1299 cells with NTF4 knockdown (Figure 4(a)). Compared with NSCLC cells with NTF4 knockdown, those with coknockdown of NTF4 and FOXL1 had higher viability, migratory cell number, and wound closure percentage (Figures 4(b)–4(d)). It is concluded that the inhibited proliferative and migratory rates in NSCLC cells with NTF4 knockdown were reversed by coknockdown of FOXL1.

## 4. Discussion

The incidence and mortality of NSCLC are both in the first place of malignant tumors [1–3]. Lung squamous cell carcinoma used to be the major histological subtype of NSCLC. In recent years, the incidence of lung adenocarcinoma has annually increased [4, 5]. A series of novel medical technologies have improved therapeutic efficacies of NSCLC to a certain degree. Nevertheless, the 5-year survival of NSCLC remains far away from satisfactory [6]. Invasiveness and metastasis are the leading risk factors for the poor prognosis of NSCLC [7, 8]. It is of significance to deeply clarify the molecular mechanisms underlying NSCLC progression.

Effective biomarkers for diagnosis of NSCLC and prediction of cancer metastasis are lacking [15, 16]. Here, a differential level of NTF4 was identified, which was upregulated in NSCLC tissues more than adjacent normal ones. We believed that NTF4 could be an oncogene involved in NSCLC.

Tumorigenesis and tumor progression involve biological characteristic changes, including persistent proliferation, apoptosis blockage, and strengthened invasiveness [17, 18]. Differentially expressed NTF4 is previously reported in many types of tumors [9, 11–13]. Our results demonstrated that knockdown of NTF4 markedly attenuated proliferative and migratory abilities in A549 and H1299 cells.

Bioinformatic prediction suggested an interaction between FOXL1 and NTF4. Later, we confirmed their binding relationship through a dual-luciferase reporter assay. FOXL1 is a transcription factor that is expressed in gastrointestinal mesenchymal cells. It is responsible for regulating tumor cell phenotypes via activating the Wnt signaling through upregulating LRP5 [19, 20]. In the present study, FOXL1 was lowly expressed in NSCLC tissues. Notably, knockdown of FOXL1 could abolish the regulatory effects of NTF4 knockdown on malignant phenotypes of NSCLC. To sum up, NTF4 was an oncogene that triggered NSCLC to proliferate and migrate through negatively regulating FOXL1. The novelty of this current study was that it was the first attempt to explore the role of NTF4 and to further investigate the potential molecular mechanism in NSCLC. However, there are still several shortages of our study. The lack of in vivo animal studies weakened the evidence level. We plan to perform tumor formation experiments in nude mice to explore the role of NTF4 in the tumor growth of NSCLC in the future. Also, we will expand the clinical sample size and prolong the follow-up to study the value of NTF4 in the prediction of patients' survival and prognosis.

## 5. Conclusions

NTF4 triggers NSCLC to proliferate and migrate via negatively regulating FOXL1. The results of the current study may provide new insights for the treatment of NSCLC.

## Figures and Tables

**Figure 1:** NTF4 was highly expressed in NSCLC. (a)-(b) Differential levels of NTF4 in NSCLC and adjacent normal tissues. (c) NTF4 levels in NSCLC cell lines. ^*∗*^*P* < 0.05, ^*∗∗∗*^*P* < 0.001. NS, no significance.

**Figure 2:** Knockdown of NTF4 reduced proliferative and migratory rates in NSCLC. (a) Transfection efficacy of sh-NTF4 in A549 and H1299 cells; (b)-(c) Viability in A549 and H1299 cells regulated by NTF4. (d) Migration in A549 and H1299 cells regulated by NTF4. (e) Wound closure in A549 and H1299 cells regulated by NTF4. ^*∗*^*P* < 0.05, ^*∗∗*^*P* < 0.01.

**Figure 3:** NTF4 targeted the regulation of FOXL1. (a) FOXL1 predicted to be a target gene of NTF4 by bioinformatic. (b)-(c) FOXL1 confirmed to be a target gene of NTF4 by dual-luciferase reporter assay. (d)-(e) Differential levels of FOXL1 in NSCLC and adjacent normal tissues; ^*∗∗*^*P* < 0.01, ^*∗∗∗*^*P* < 0.001.

**Figure 4:** NTF4-regulated NSCLC cell phenotypes by negatively regulating FOXL1. (a) Transfection efficacy of sh-FOXL1 in A549 and H1299 cells. (b) Viability in A549 and H1299 cells coregulated by NTF4 and FOXL1. (c) Migration in A549 and H1299 cells coregulated by NTF4 and FOXL1. (d) Wound closure in A549 and H1299 cells coregulated by NTF4 and FOXL1. ^*∗*^*P* < 0.05, ^*∗∗*^*P* < 0.01.

## Data Availability

The datasets used and analyzed during the current study are available from the corresponding author upon request.
